# Research on Geriatric Care for Equalizing the Topological Layout of Health Care Infrastructure Networks

**DOI:** 10.1155/2021/8306479

**Published:** 2021-05-26

**Authors:** Rui Liu, Miao Du, Jun Shen, Xiaolan Wang, Ying Jiang

**Affiliations:** Shanghai University of Medicine & Health Sciences, Shanghai 201318, China

## Abstract

In this paper, through the study of elderly care, the method of equalizing the topological layout of the health care infrastructure network is used for in-depth analysis. With the evaluation method of senior care facility fairness as the research base theory, the analysis and evaluation of senior care facilities are carried out from two aspects of supply and demand fairness and spatial fairness, and the problems and shortcomings of senior care facilities in terms of facility scale, spatial layout, service level, and policy management are summarized. This paper analyses the contradictory points of the nonequitable layout of urban senior care facilities, to propose planning suggestions and optimization measures for the planning of the senior care service facility system. It discusses the problems in the spatial layout of senior care facilities from the perspective of social equity, focuses on the needs of urban disadvantaged groups, promotes the equalization of public services, and provides the theoretical basis and technical support for the planning policy of urban public service facilities. The study fully combines the theory of urban planning disciplines with geographic information system technology, mathematical and statistical technology, and network data acquisition technology to establish the evaluation of the spatial layout of senior care facilities based on social equity framework, to contribute to the planning of similar urban public service facilities. It comes to make an integrated consideration of the supply content and scope of basic public service facilities and check the gaps, which is conducive to improving the scientific and intensive nature of public resource input according to local conditions and more speed and provides some reference to the method of public service facility allocation.

## 1. Introduction

Whether the supply and demand of urban senior care facilities are balanced directly affects the efficient use of public service resources, which in turn directly affects the fairness of urban residents' access to urban public services. The attractiveness of living space to people is multiplied by the positive externalities of senior care service facilities, and urban senior care facilities are highly clustered locally or in specific areas due to the differences in living space, resulting in the uneven spatial distribution of senior care facility resources and uneven guarantee of senior care services among different social groups, which generates the phenomenon of polarization of facility layout [1]. The aging society is facing the contradiction of a large and fast-growing elderly population, while the total supply of elderly services is insufficient and unevenly distributed in space. This has resulted in a polarization of the layout of facilities, with a surplus of facilities in rich areas and a lack of facilities in disadvantaged areas. Therefore, it is necessary to introduce the perspective of social equity in the evaluation of urban senior care facilities, which not only is helpful to efficiently promote the achievement of planning objectives but also can help to better improve the content of planning, to find the solution to the problem according to the evaluation results, which is important for the rationality of planning, the fairness of facility layout, and the real sense of realizing the function of public policy of urban planning. It is important for the rationalization of planning, the fairness of facility layout, and the real realization of the public policy function of urban planning [2].

Based on the current social development and the current situation of senior care facilities, the shortcomings of the traditional senior care model have gradually emerged, and although senior care facilities have become an important supplement to senior care, there are indeed many defects in their development [3]. This paper explores the path of constructing a fairness evaluation method for urban senior care facilities based on the perspective of social equity, compares the current situation of senior care, discusses and summarizes the supply and demand equity and spatial equity of senior care facilities, and provides planning strategies and feasible opinions for senior care facilities to create a better life for the elderly [4]. The study comprehensively evaluates the social equity of the layout of senior care facilities, explores the current layout problems, and carries out a systematic and multi-dimensional comprehensive analysis of the layout of senior care facilities through geographic information technology, web crawler analysis technology, and mathematical statistics technology. As an especially disadvantaged group, elderly people have the characteristics of small activity range and low physical ability, etc. The study starts from the attributes of elderly people, fully considers their living needs, analyses the characteristics of their economic and social attributes, analyses the fairness of urban elderly facilities with the Gini coefficient and Lorenz curve as the research methods, and establishes a social fairness-oriented theoretical framework that can provide theoretical ideas for the fairness of other facilities [5]. The study provides some research ideas to help the elderly to live happily and enjoy their old age. Community management is the basic content of urban management, while community service is an important part of community management and is the external manifestation of community management. With the development of socialist market economy, the demand for community services from most residents has become increasingly diversified and the requirements for community services have become higher and higher. With the advancement of urbanization and social development changes, the community services of the old communities built in the era of planned economy can no longer meet the basic needs of residents. This paper analyses the current situation of community services in *N* communities, discusses the problems of community service construction, and proposes countermeasures and suggestions for community service construction according to local conditions.

The maximum value realization of urban public services is related to not only the content of the services themselves but also the effective spatial allocation of the corresponding facilities. Then, the spatial distribution and scale configuration of public service facilities at different levels will directly affect the equalization and fairness of public service facilities. Between regions and urban and rural areas, people pursue parity, including public services and basic protection that everyone can enjoy, and everyone's basic rights and interests can be respected and can develop freely, etc. While emphasizing fairness, spatial justice also focuses on efficiency and pursues the realization of holistic and long-term benefits. Promoting the equalization of basic public services is an important manifestation of spatial justice in social development, such as public medical services, building a multi-level medical and health care system covering urban and rural areas, improving the coverage of medical insurance, and guaranteeing the medical needs of residents. In this context, the connotation of spatial justice theory has been deepened and the application field has become more and more extensive.

## 2. Related Work

In general, foreign developed countries inevitably must go through three different stages of development, i.e., the traditional life care institution stage, the nursing institution stage, and the community care institution stage, etc. [6]. There are three trends in the choice of elderly care models in developed countries: the “home-based elderly care” model in which the family is the unit for elderly care, the “home-based elderly care + institutional elderly care” model in which the family is the main unit for elderly care and institutional care is supplementary, and the “community care home-based elderly care + institutional elderly care” model in which “collective elderly care is the concept” [7]. According to Guo et al., the needs of the elderly are an important criterion for planning the location of elderly care facilities, and the level of service, care capacity, and communication space greatly influence the direction of elderly care facilities planning [8]. The needs of the elderly are an important criterion for the planning of elderly facilities, and the level of service, care capacity, and communication space greatly influence the direction of elderly facilities planning [9]. By analysing the construction mode and service approach of day-care facilities for the elderly in the UK, Di Nardo et al. concluded that the layout of elderly facilities needs to rely on community service centres, community elderly service facilities, community hospitals, and other community public service facilities, and the structure of the facilities should be based on the core of the dining room or activity room, with several segments of basic services, recreation and leisure, personal care, and medical rehabilitation according to the nature of different services [10].

Ngowi constructed a multi-objective school siting decision model that includes the risk of tsunami hazard to the plot, the sum of transportation cost of students to school, the school service area under a certain threshold, and the construction cost from the practical problem of sitting elementary school in tsunami-prone areas of Sri Lanka and used a non-dominated ranking genetic algorithm to obtain the siting results [11]. In their study, Dr. Shabbir et al. analysed the historical characteristics of the development of population aging and the characteristics of elderly care in different historical stages [12]. Neighbourhood mutual aid networks are built based on geography, with the government providing economic and policy support and volunteers and social groups providing elderly care services, targeting mainly the elderly living alone and the disabled [13]. The frequent interactions between members and their trusting acquaintance create convenient conditions and a harmonious atmosphere for the development of mutual aid [14]. In addition to taking care of the elderly in a mutual help and self-help way, the network also carries out various hobby activities such as swimming, fitness, and dinner and popularizes the knowledge and skills of health care in the process to improve the self-help ability of the elderly [15]. Neighbourhood mutual aid network not only plays a positive role in reconstructing the interpersonal network of the community but also creates opportunities for widows, widowers, and senior citizens to communicate with the outside world, providing a platform to share the joy of life, relieve the misery, and maintain an optimistic and open-minded attitude, helping the elderly to spend their old age positively and optimistically.

At the theoretical level, there are a lot of research results on neighbourhood centres and living circles, and the distribution of the fields is relatively wide. As different models of community service support, both have their advantages and values, but there is a general lack of understanding of the multiple connotations of neighbourhood centres and living circles, and there is a gap in the comparative study of the two models. Based on the public service needs of the elderly population and data acquisition, we selected relevant indicators and established the “15-minute living circle” public service evaluation index for the elderly population aging in place, used the population spatialization grid data to generate the community population centre of gravity, and used web crawler technology to obtain the walking traffic cost data. Based on these data, the “15-minute living circle” scope of the community is generated to evaluate the distribution of public services in the main urban area, identify the weak points, and provide a better basis for the spatial layout and planning of urban elderly care services.

## 3. Analysis of Health Care Infrastructure Network Topology Layout Equalization for Geriatric Care

### 3.1. Equalization Analysis of Medical Facility Network Topology Layout

Urban senior care facilities are the spatial carriers of social senior care services, which need to have a fixed place environment in urban space. At the same time, it also needs a certain amount of space to be equipped with the relevant teams and materials for the elderly service to ensure the user experience, such as medical teams and rehabilitation places and catering teams and dining places. Thus, the spatial entities of urban senior care facilities exist in the urban space in the form of points, with fixed locations and scattered layouts, and users need to overcome spatial barriers through transportation carriers to access the service resources of senior care facilities [16]. As the core issue of urban government functions, the degree of perfection and meaningfulness of public services not only consider the government's ability to solve people's livelihood problems, but also reveal the value of government administration. Therefore, the purpose and significance of studying the value of urban public services are to correct the livelihood orientation of government public services; to clarify the value criteria for selecting, judging, positioning, and evaluating the governing behavior and activities of urban governments; to shape the value ideal of urban government public services; and to reveal the value pursuit of urban government public services. Urbanization brings relatively concentrated resources and values to urban centres, which means that urban centres have absolute advantages in terms of location and resources, attracting urban residents to migrate to the centres. The migration of population raises the demand for housing in the central area, resulting in higher land value and higher development intensity, and the central area gradually becomes a business centre. The construction of urban elderly facilities is developing slowly, and in the process of urban spatial differentiation, they are often squeezed by functional blocks with better market efficiency. As a result, urban elderly facilities tend to be small in volume and large in number in densely populated central areas and large in volume and small in less densely populated areas, thus forming a phenomenon that the distribution of elderly facilities cannot be coupled with the distribution of the applicable population.

The mobility of UAVs causes the distance between any two nodes in FANETs to vary with time, and the conventional interference model can only obtain the cumulative interference value at time *t* (called the instantaneous interference value) [17], which does not accurately reflect the current channel state. Also, the fast mobility makes it very difficult for the UAV to obtain the state information of all channels, and the instantaneous interference value can only reflect the current channel state, so it is necessary to find a method that can satisfy the variation of the distance between nodes and accurately reflect the current channel state. The interference prediction method satisfies the requirement well by calculating the average interference value in time *t* based on the node's movement model using the integration idea.

(1) $$\begin{array}{c} E\left[I_{j}\left(t|t_{0}\right)\right]=\sum_{i,j}\frac{1}{\Delta t}\int_{I_{0}}^{I}g_{ik}\left(y^{i}\left(t\right)\right)\cdot f_{y}\left(y^{j}\left(t\right)\right)\text{d}t. \end{array}$$

Using equation (1), the Signal-Interference Noise Ratio (SINR) at node *j* can be obtained.

(2) $$\begin{array}{c} \kappa_{j}^{i}\left(t|t_{0}\right)=\frac{\sum_{i,j}\left(1/\Delta t\right)\int_{I_{0}}^{I}g_{ik}^{\Delta t}\left(y^{i}\left(t\right)\right)\cdot f_{y}\left(y^{j}\left(t\right)\right)\text{d}t}{N_{0}+E\left[I_{j}\left(t|t_{0}\right)\right]}, \end{array}$$

where *N* denotes the ambient noise variance, which is generally set as a constant. According to equation (2), the average link capacity in interval *t* can be obtained.

Public goods theory is a basic theory of the new political economy, which mainly studies how to properly deal with the relationship between the government and the market and how to transfer the history of government functions, such as Home, Samuelson services marketization, and other issues. Lindahl has made outstanding contributions to the development of public goods theory; public goods have three outstanding characteristics: the indivisibility of utility, non-exclusivity of benefit, and non-competitive consumption, compared with private goods, have distinctive opposing characteristics [18]. Medical services are essentially public goods, and their service targets and beneficiaries are citizens. The government and the market should improve and balance the service quality of medical facilities. The government plays a vital role in changing the quality of medical services. The local medical level should be improved to provide high-quality medical services for public welfare and to ensure the sound operation of service facilities. How to ensure that people enjoy high-quality medical services for public welfare is a hot research topic, as shown in Figure 1.

Based on the service scope requirement of reasonable accessibility, to meet the public service facility configuration requirements of urban and rural integrated development, it is also necessary to pay attention to the efficiency of the use of supporting facilities. The research basis of the thesis is to make public service facilities meet the configuration requirements of urban and rural areas through the residents' demand for public service facility configuration, and to meet the living needs of internal residents, thus enabling to improve the service efficiency of the whole facility system. To facilitate the allocation and assessment of resources, the administration usually classifies the resources into uniform standards and sets the corresponding standards, which can be based on the theory of planned economic management and can be inherited and is feasible in practice. The elderly, on the other hand, generally do not dare to easily purchase their own medication for treatment when they are sick, but will take the initiative to seek medical treatment. Since the financial transfer payment mechanism to hospitals is not yet perfect under the current medical system, there is a serious information asymmetry between doctors and patients, and medical professionals tend to use their information advantage to prescribe mid-to high-end drugs to patients to boost their own income. This makes medical consumption in the city tend to favour the middle and high level of medical consumption. However, it cannot keep pace with the development of urbanization, nor can it meet the needs of the residents, nor can it enrich and improve the level of services based on the changes of the residents' facilities and life. The optimal configuration of public service facilities should be based on social reality and human-oriented thinking, and the social attributes of service settings should be incorporated into the spatial layout to make it more humane in the process of use.

(3) $$\begin{array}{c} C_{ij}=W\log\left(20+\kappa_{j}^{i}\left(t|t_{0}\right)\right),\\ P_{ij}^{ON1}=1-e^{\left(-\left(5^{r_{ij}}-1/s^{i}\right)\right)}. \end{array}$$

The size of each packet is assumed to obey an exponential distribution with a mean value of *K* bits. Each node maintains a single queue and delivers the packets to the relay nodes according to the first-come-first-served principle. According to the conclusions obtained in [19, 20], when the arrival process obeys a Poisson distribution and the service process obeys an independent exponential distribution, the average delay of links *i*, *j* at time *t* can be approximated as

(4) $$\begin{array}{c} M_{ij}=\frac{24\kappa }{C_{ij}-r_{ij}}. \end{array}$$

The elderly service function is the characteristic attribute of the elderly facilities, and different service contents and forms of action are generated by different service functions of various facilities, which in turn clarify the service targets, service scope, and spatial level. The senior care service system under the concept of mutual aid senior care should be based on the principles of “continuous care” and “precise configuration” to provide precise and applicable senior care services for the elderly with different physical conditions and different senior care needs. As a spatial entity, senior care facilities need to be built and landed, so the support of space and environment is indispensable. The site selection and spatial layout of various facilities should take full consideration of the building environment and its surrounding influencing elements, and the physical construction should be carried out in an orderly manner under the condition that the environment meets the construction conditions. The construction of senior care facilities under the concept of mutual aid senior care should consider the undertaking with the mutual aid senior care mode and meet the requirements of use. The input supply of the facility determines the starting point and height of the facility construction, and the implementation of the construction determines the input-output efficiency and the actual supply efficiency of the facility. In the past, the supply of rural public products depended on the government's financial allocation and villagers' self-financing, and the pressure of local finance and limited rural economy led to the limited capital investment in rural senior care facilities. Therefore, under the concept of mutual aid elderly care, the main body of input supply should be innovated to improve the input-output efficiency and guarantee the level and quality of facility construction on the ground, as shown in Figure 2.

The planning, construction, and management of senior care facilities belong to the category of public facilities, which are subject to the supervision and control of several government departments. The management and operation of the facilities after the completion of construction is related to whether the facilities can be used normally and whether the senior care services can be provided. According to the public facility operating body, senior care facilities can be divided into public-run, privately run, public-private, and privately run public facilities, etc. The mutual aid senior care facilities studied in this paper have public welfare attributes, and their management and operation methods need to be innovated to maintain the normal use and operation of the facilities. The elderly care facilities under the concept of mutual aid are different from the traditional elderly care facilities in that the elderly care service mainly relies on the mutual care and companionship among the elderly and the voluntary service of social forces, and the service quality is more subject to the maintenance of emotion, responsibility, and morality, which is unstable. The first benefit is that decentralized uniformity can reasonably save resources, the second benefit is that all can get the service they deserve, and the third benefit is that the quality of the service can be maximized. Therefore, it is necessary to establish institutional guarantee in the actual operation process and properly handle the relationship between emotion and system to ensure the quality of mutual-aid elderly care service level.

From the previous review of the planning research on neighbourhood centres and living circles, it can be seen that the research results of the two studies show different orientations: the research on neighbourhood centres mainly explores several aspects of the neighbourhood centre model, public service facility configuration and community business model, pointing to the supply side of public or commercial services such as government, public sector, and market, while the research on living circles mainly explores several aspects of territorial spatial structure. Although it also points to the supply side, using the circle of life as the theoretical basis means that the research is conducted from the demand side, representing the interests of residents. This orientation also echoes the transformation direction of residential planning-“people-oriented” as the core, community life circle planning oriented to life services. Therefore, the author believes that the neighbourhood centre model can correspond to the supply side and the living circle model to the demand side.

If equations (5) and (6) are established, the receive operation starts to receive partition information from the main process and initializes the subregion flow field.

(5) $$\begin{array}{c} D_{1}=w_{11}x_{1}+2w_{12}x_{2}+4w_{13}x_{3}, \end{array}$$

(6) $$\begin{array}{c} D_{2}=w_{21}x_{1}+2w_{22}x_{2}+4w_{23}x_{3}. \end{array}$$

Continuing with the unfinished calculations, the received operational flow field is counted to obtain

(7) $$\begin{array}{c} V\left(i,j\right)=\sum_{m,n}I\left(i+m-2,j+n+1\right)\cdot K\left(m-1,n+1\right). \end{array}$$

It was found that the activity preferences of different older people in rural areas in southern Jiangsu showed common characteristics and individual differences. In terms of common characteristics, we found that most of the elderly in rural areas prefer to gather and communicate in crowded places, tend to do activities according to their interests and preferences, and show a higher enthusiasm for interaction than middle-aged people, and show a preference for solitude in semi-public spaces due to their questioning and resistance to external things. In terms of individual differences, it was learned during the visit that the elderly in rural areas of southern Sudan would keep working and insist on self-support as long as they were healthy, and their conditions permitted. The purpose of the study is to maximize the homogeneity of public service areas and populations, and to provide people with the most equal access to services. In the survey on daily activities, most of the elderly still need to do housework, farming, and other physical labour; daily leisure activities are mainly focused on watching TV, planting flowers, board games, and chatting, and cultural and recreational activities are relatively monotonous. Many villages have organized relatively good cultural and recreational activities, but the elderly also expressed little interest.

### 3.2. Geriatric Care Design

The family model of elderly care based on blood ethics has a long history, where children are the main providers of resource support for elderly care, responsible for the elderly's food, living, and spiritual care. The economic and social characteristics of the countryside dictate that elderly people rely mainly on their children to solve their senior care needs, which is one of the factors that most elderly people choose to age in the family. During the research, it was found that the elderly interviewed were most concerned about two major issues: the first was the difficulty in taking care of themselves due to old age and declining physical functions; the second was that the elderly were mostly worried about the difficulty in getting timely medical treatment when no one was around in case of physical emergencies or emergencies. Some elderly people say that they have limited daily communication partners and monotonous leisure activities, and they are often lonely and despondent. All in all, the needs of senior care, health protection, and spirituality in the family aging method are highlighted. The reason for this is that the population in rural areas of southern Jiangsu is very mobile, and the number of empty nesters is gradually increasing as the family structure becomes smaller and more “nucleated,” and the spatial distance makes it more difficult for children to take care of the elderly, and the traditional intergenerational support model is changing. The traditional intergenerational support model has changed and the support from children has weakened, making it difficult to guarantee the quality of elderly care in rural families. Empty nest families and elderly people living alone are more likely to have a lonely mentality, and elderly people who cannot take care of themselves without the company of their children are at risk for their health and safety.

According to the unified deployment of the district committee and the district government, the district major project office shall integrate all forces, rationally arrange functions, and coordinate the coordination, scheduling, promotion, supervision, and management of project construction services. It is necessary to adopt an effective project classification and packaging method, division of labor and responsibility, and step-by-step implementation. Social investment, government investment, and competition for funds are three types of packaging methods for large projects. At the same time, it is necessary to coordinate the project management with the District Transportation and Urban Development Bureau, the District Water Conservancy Bureau, the District Education Bureau, and the District Commerce and Food Bureau.

The community-based elderly care model, also known as home care, where the main supply of elderly care resources in the community and the elderly live at home and receive relatively professional home care services or choose community care services, has played a good role in urban areas. However, even in the economically developed rural areas of southern Jiangsu, only 11% of the elderly people chose community aging, mainly because they could receive care without leaving their familiar living environment. The main reasons why the elderly do not prefer community-based senior care are that they can take care of themselves, they do not have time for farming, the cost, they must take care of their grandchildren, and they do not know about it because it is not very popular. In rural areas, the concept of community is different from that of modern urban communities, and the organization and construction of a community-based senior care model are still in their infancy in rural areas. Factors such as limited resource conditions, lack of professional caregivers, capital and facilities, and the fact that an efficient management system has not yet been established all make the community-based elderly care model currently unavailable in rural areas of Southern Sudan, as shown in Figure 3.

All-age livable communities are urban communities for all people of all ages to live in and live in for life. It is different from traditional urban retirement communities that isolate the elderly as a special group, but treats them equally as people of other ages, thus achieving the development of integrated social intergenerational relationships. The intergenerational relationship usually refers to the interpersonal relationship between the elderly and young people, which can occur both in the family and within the society. The development of intergenerational groups, such as the elderly and young people, is often fragmented, and the increasing miniaturization of family size makes it difficult to meet the needs of intergenerational emotional exchange, knowledge exchange, and life assistance. Localized senior care facilities should take up the social responsibility of building an all-age living environment in the community while focusing on the care of the elderly.

In line with the construction concept of integration with urban communities, setting up a regional exchange space within a regionalized senior living facility creates opportunities for people from different generations to meet and communicate. The elderly in the community not only act as a one-way care recipient but also share their life experience and skills with other groups such as young people and children. As with the German “multigenerational house” concept, many retired seniors in the community have expressed their willingness to serve other intergenerational groups who join the facility on a voluntary and pro bono basis, and youth groups in the community are willing to participate in the “multigenerational house” program. First, it is close to public spaces and soft partitioning. This allows for a large open space that can accommodate all the elderly in the facility to organize large events. Secondly, it is combined with the public space. In the case of limited public space, it can be combined with the dining room, rehabilitation training area, or unit living room to achieve multi-functional use of space and more efficient facility management. Separate from other public spaces of the facility, it has the least impact on the normal operation of other functions, as shown in Figure 4.

The elderly in the community can enjoy health management services at the community health service centre where they live, specifically involving free health check-ups (including general physical and auxiliary examinations), lifestyle and health status assessments, and the resulting establishment of a network health file [21]. At the same time, the territorialized elderly facilities implanted in the community can also collect various types of information on the elderly in the community containing their health status, economic status, living condition, and willingness to provide elderly services while providing services. On this basis, both parties can further improve the information within the community health management platform for the elderly. Based on the real-time access to the health status of the elderly in the management platform, the community primary medical institutions can make reasonable and effective treatment plans for them, and enable the elderly to detect diseases early and carry out treatment early, to prevent the development of diseases and reduce the disability and death rates; after obtaining the health records of the elderly provided by the community health service centre, the elderly facilities can also use them to guide and optimize the facilities' care services for the elderly. The health records provided by community health service centres can also be used to guide and optimize the content of care services tailored to individual elderly people, thus improving the accuracy of service positioning and the economy of operating costs.

Most of the existing buildings have a series of problems such as poor structural stability, the mismatch between the existing structure and new functional use, and limitation of transformation diversity due to age and disrepair, failure to consider future transformation flexibility at the beginning of construction, and other factors. Therefore, the main structure optimization should be implemented based on the overall composite seismic performance of the reinforcement treatment, mainly using the paste steel plate (steel components) and other dry construction methods for seismic reinforcement. The principle of paste steel plate reinforcement method is to use adhesive to paste the steel plate on the surface of the original member so that the steel plate and the original structure form a new bearing system, and the steel plate is involved in the force, to achieve the purpose of reinforcing the concrete structure. Due to the development level of rural areas in southern Jiangsu and the traditional concept of rural elderly people, community and institutional retirement are usually not widely recognized and accepted by rural elderly people and are usually not the ideal choice. With the continuous population migration, the population structure will gradually evolve towards advanced aging, and the situation will be more severe. The economic and social conditions and the construction level of rural areas in southern Jiangsu are limited, and their elderly care foundation is relatively weak. It is imperative to innovate the elderly care model and explore new paths for elderly care in the current context. The mutual help elderly care model has been explored in different forms in different parts, and the current development is widely accepted by the elderly and their families, and the development trend is good, which is an effective elderly care model.

## 4. Analysis of Results

The level of construction of community service support is significantly related to the region. Old urban areas have been built for a long time, and the development of various service facilities is relatively complete, while new urban areas and urban fringe areas are lagging in the construction of service support due to factors such as short construction time and distance from the city centre. Therefore, no matter from the total score of community services in each region or the score of public and commercial services in each region, the old city communities are far more than the communities in the other two types of regions in terms of score. However, through field research and visits, it is found that the old city also has problems such as overpopulation, shortage of land, the aging physical environment of service facilities, and limited space for landing and expansion of new service facilities, as shown in Figure 5.

However, at the same time, the living space differentiation makes the shared use of service facilities a major difficulty. For example, commercial houses are located close to urban villages, and commercial houses adopt fully closed management, so the service facilities located inside the community are only open for use by the residents of the community, which is not conducive to improving the efficiency of the facility utilization, increasing the difficulty and pressure of facility supply, and even easily sowing the hidden danger of social differentiation. Moreover, the large scale of the neighbourhood is also the reason for the lack of sharing of community service facilities, such as the closed neighbourhoods in the form of commercial houses. The large scale of the neighbourhood means that there is not enough space for roads and alleys, and there is a lack of space for service facilities, especially commercial service facilities, and the service facilities are clustered in blocks to form small-scale service circles, and the service scope only involves the surrounding small-scale residential areas. However, according to the research and interviews, it has the problem of attaching importance to the construction of street-level facilities but not enough community-level facilities. The number of facilities within the boundary is much higher than the number of facilities within the community. The community-level facilities can better take care of the needs of the elderly, children, the disabled, and other disadvantaged groups for short-time travel and convenient use, better meet the sense of service access and experience of community residents, and are more conducive to service sharing and neighbourhood construction within the community. Therefore, it is necessary to focus on the construction of community-level service facilities in the hierarchical setting of service facilities.

As Figure 6 shows the evaluation chart, unlike other public service facilities, in the East Lake Scenic Area, the community coverage rate of parks and green squares and the coverage rate of the elderly population both reach 100%, and the elderly population has sufficient space for activities. Also, the highest area only reached 73.80% and 75.70%, while the lowest area, Jingkai, only reached 38.46% and 59.68%, leaving much room for improvement. Development coordination index: there are five zones higher than 1, including 1.36 points in the East Lake Scenic Area zone, and the lowest 0.36 in the Jingkai zone. The overall imbalance index is 3.95, which is the lowest among all facilities because each park green space in the East Lake Scenic Area covers a larger area, but there are not many of them, so the gap is not widened.

From a horizontal perspective, summarizing the basic data of each street, extra-large senior care facilities can serve only 4 settlements, and small and medium-sized senior care facilities can serve 19 and 18 settlements, respectively, which shows that the distribution equity of extra-large senior care facilities is the worst; through the visualization results, we can find that extra-large senior care facilities provide a large amount of effective service area of senior care facilities for the settlements they serve, thus with the settlements that cannot be served. There is a huge quantitative difference; medium-sized senior care facilities provide the widest service coverage for the region, with 50% of the residences being served by more than half of the effective service area of medium-sized senior care facilities; small senior care service facilities provide relatively fewer services overall, but in some residences, they perform better in terms of the effective service area provided compared to medium-sized senior care facilities. The remaining settlements have one or two types of facilities to choose from, as shown in Figure 7. Among them, the residents of Hexing Road Street have the highest service area per capita of 19.22 m^2^/person, while the residents in Lujia Street have the lowest, with only 1.06 m^2^/person.

At the same time, it is suggested that the centrally located facilities can improve the accessibility of senior care services through door-to-door mutual aid services, improved transportation conditions, and shuttle bus transportation services so that the senior care services in administrative villages can radiate to natural villages and natural village senior care services can radiate to residential groups, forming a full-coverage network system of rural senior care facilities, especially for the aging villages where the land is sparse; this way can effectively expand the coverage of senior care facilities. Establishing a comprehensive mechanism for expressing social interests and guiding the masses to express their interest demands in a rational and legal form is the primary link to improve the coordination mechanism for social interests. To establish a perfect mechanism for expressing interests, it is necessary to give full play to the functions of existing channels for expressing interests and to open new channels for expressing interests according to the development and changes of interest groups. The coverage area of senior care facilities can be effectively expanded, especially for the aging villages with sparse land. The spatial layout of senior care facilities under the concept of mutual aid senior care should be flexible and precise and should not be limited to the establishment of a standard system but should take the integration with actual needs as the first factor. Rural areas can be flexibly laid out and set up under the premise of satisfying the site selection requirements and the needs of the elderly and the reasonable use of resources. The following are some suggestions for the layout of administrative villages, natural villages, and residential groups for elderly facilities, as shown in Figure 8.

Also, cultivating a free and democratic social atmosphere and constructing a perfect interest expression and feedback mechanism in the current urban-rural context can help strengthen the basic right to survival and development of rural residents, as well as improve the human living environment, maintain social stability, and guarantee the rational political participation of villagers. The available rural locations have many options and are also less expensive compared to urban areas, so they are easier to layout. Guiding rural residents to rationally and accurately express their actual needs, give feedback on the effectiveness of construction, and expand the depth and breadth of public participation can not only assist the government in strengthening the accuracy of decision-making, but also help alleviate social conflicts, coordinate the balance of interests, and stimulate rural residents' enthusiasm to participate in the construction and enhancement of public utilities, as well as promote the development of rural planning and construction in a scientific and rational direction. In terms of configuration standards, a flexible and adaptable allocation standard system is proposed for the use characteristics of various types of elderly facilities, optimizing the “one-size-fits-all” mechanical allocation means and making up for the gaps in the basis for the allocation of elderly facilities. In terms of spatial layout, it breaks the solidified idea of centralized layout mode and adopts the embedded layout mode of “large centralized and small scattered,” which improves the effective coverage and service accessibility of the facilities and creates convenient conditions for the elderly to use. In terms of mechanism guarantee, the innovative organization and operation mechanism expands the sources of support for the elderly, relieving the pressure of the government's one-dollar supply and the dilemma of the weak rural elderly foundation; by improving the interest expression and feedback mechanism, the interaction between the villagers and the government and the planners and builders is promoted, and the accuracy of the facility supply and the timeliness of the feedback of the construction effectiveness is enhanced; by establishing the information management service platform, the comprehensive elderly care cost is reduced and the level of the facility service and management is improved. At the same time, it improves the service level, management efficiency, and supervision of the facilities.

## 5. Conclusion

There are certain correlations and differences in planning research and planning practice, and both are important as models of community service support in terms of their supply and demand. Neighbourhood centres and living circles hold different positions. Neighbourhood centres are a coordinated means for planning elites, city managers, and service providers to provide quality public and commercial services to urban communities, and their paths are top-down planning conduction, focusing more on the supply side; living circles, on the other hand, are concepts introduced into the planning community from geography, which are essentially behavioural space planning, and the subject of behavioural activities is people. The core of the living circle model is people-oriented, starting from the daily activities and living needs of urban residents, and its path is a bottom-up expression of demands, with more emphasis on the demand side. The construction mode of the “new neighbourhood centre” needs to clarify the new characteristics of the neighbourhood centre in the context of the living circle, and there is an interactive relationship between the neighbourhood centre and the living circle. The connotation and scope of application of the new neighbourhood centre have been expanded. Neighbourhood centres can organize spatial elements in an integrated manner and become a platform or carrier for the coordination and co-construction of multiple parties; adopting a differentiated spatial organization and construction mode, neighbourhood centres adopt a mixed, composite, and shared spatial organization, corresponding to “functional building clusters,” “one-stop complexes,” “one-stop complexes,” “one-stop complexes,” and “one-stop complexes.” The construction modes of “one-stop complex” and “embedded service space” are adopted; diverse types of functional combinations are adopted, such as medical and health care, cultural and sports, commercial, comprehensive, and innovative neighbourhood centres.

## Figures and Tables

**Figure 1:** Network topology layout design of medical facilities.

**Figure 2:** Trends in population change.

**Figure 3:** Distribution of reasons for old-age maintenance.

**Figure 4:** Construction of network information platform for senior care facilities.

**Figure 5:** Total score of community service support by region.

**Figure 6:** Coverage and coordination statistics.

**Figure 7:** Distribution of effective service area of each level of elderly facilities on a street scale.

**Figure 8:** Changes in spatial layout distribution.

## Data Availability

Data sharing is not applicable to this article as no datasets were generated or analysed during the current study.
